# Primary Exploration of Efficacy of Community-Family Management Mode under Internet-Based Mobile Terminal Monitoring in Elderly Patients with Stable Coronary Heart Disease

**DOI:** 10.1155/2022/7043928

**Published:** 2022-01-25

**Authors:** Xiang Li, Wenwu Zheng, Jinsong Li, Yibin Gao, Qiang Lin, Jinfeng Yang, Shuiying Huang, Defang Wang, Bin Wang

**Affiliations:** ^1^Department of Cardiology, Luzhou People's Hospital, Luzhou City 646000, Sichuan Province, China; ^2^Department of Cardiology, The Affiliated Hospital of Southwest Medical University, Luzhou City 030699, Sichuan Province, China

## Abstract

**Objective:**

To explore the efficacy of community-family management mode under Internet-based mobile terminal (MT) monitoring in stable coronary heart disease (CHD) in the elderly.

**Methods:**

A total of 86 patients with stable CHD treated in our hospital from May 2018 to May 2021 were selected as the study objects for the retrospective study and were divided into the control group (routine intervention) and the research group (community-family management mode intervention under Internet MT monitoring) according to the health management modes, with 43 cases each, and the health behaviors and control of CHD were compared between the two groups.

**Results:**

No statistical between-group differences in general information were observed (*P* > 0.05); 6 months after intervention, the control of laboratory indexes including blood pressure, blood glucose, triglyceride, and total cholesterol in patients was obviously better in the research group than in the control group (*P* > 0.05); after intervention, the scores on rehabilitation knowledge level and secondary prevention behavior were obviously higher in the research group than in the control group (*P* > 0.05); 6 months after intervention, the scores on physical limitation, anginal stabilization, anginal frequency, disease perception, and treatment satisfaction were obviously higher in the research group than in the control group (*P* > 0.05); compared with the control group within 1 year of intervention, the readmission rate of the research group was significantly lower (*P* > 0.05); and compared with the control group, the total score of CQQC and scores on physical strength, condition, general life, and social mentality were significantly better in the research group (*P* > 0.05).

**Conclusion:**

Community-family management mode under Internet-based MT monitoring is the valid continuation of clinical nursing for elderly patients with stable CHD, which plays an effective role in terms of daily monitoring indexes, stabilizing condition, improving disease cognition, reducing the readmission rate, and improving the prognostic quality of life of patients.

## 1. Introduction 

Coronary heart disease (CHD) refers to the coronary atherosclerotic heart disease whose predisposing and risk factors mainly include hypertension, blood lipid abnormality, hyperglycemia, as well as adverse lifestyle (e.g., excessive alcohol consumption, smoking, unjustified diet, and lack of exercise), and its onset is often associated with factors such as seasonal variations, physical activity, and emotional excitement [1–4]. As clinical research deepens, most patients can be effectively treated, but if a short period of rapid treatment is not accompanied by long-term and effective health management interventions, adverse risk factors can still lead to life-threatening recrudescence. Therefore, continuous nursing intervention inside and outside the hospital is very important for CHD patients. Since the issuance of the Twelfth Five-Year Plan of China on Aging Undertaking Development [5] (No. 28 document of State Council in 2011) by State Council, the gradual establishment and perfection of a continuous care delivery system where the elderly are “supported by institutions, provided with home care, and taken care of by community” has been proposed, and by establishing the “community-family management mode,” our hospital has gradually formed a continuous health management system of CHD based on clinical care, in the hope of further meeting the health service needs of elderly patients with stable CHD, reducing the readmission rate of patients, and then promoting the continuous development of nursing industry. In addition, our hospital has creatively combined the community-family management mode with the currently booming MT, expecting to promote the health management efficacy and quality with the intervention based on MT service platform for patients, with the results summarized as follows.

## 2. Study Methods

### 2.1. Case Screening

According to the study objective, the inclusion and exclusion criteria were as follows. Inclusion criteria: (1) patients met the clinical diagnosis criteria for stable CHD in Guideline for Diagnosis and Treatment of Stable Coronary Heart Disease (2018) [6] and were in the stable stage of disease, (2) patients or their family members who provided long-term care could go along with the intervention of community-family management mode under Internet MT monitoring, (3) patients had higher compliance with the continuous health education inside and outside the hospital implemented by our hospital, and (4) patients and their family members understood the study and agreed to join the study. Exclusion criteria: (1) patients had cognitive disorder or seeing-hearing disorder, (2) patients were accompanied with other severe and unstable physical illnesses, (3) critically ill CHD cases, and (4) patients' clinical data were incomplete. According to the aforesaid criteria, 86 patients with stable CHD treated in our hospital from May 2018 to May 2021 were selected as the objects for the retrospective study.

### 2.2. Case Grouping

A total of 86 patients meeting the inclusion and exclusion criteria were divided into the control group and the research group according to the health management modes; to be specific, those who received routine intervention were included in the control group, and those who accepted the community-family management mode under Internet MT monitoring were included in the research group, with 43 cases each. The study project was verified and approved by the hospital ethics committee.

### 2.3. Methods

Routine intervention: routine health education in the forms of face-to-face consultation or oral education was implemented to patients during their hospital stay, the contents mainly included health guidance on patients' condition, prevention and treatment of complications, and secondary prevention, and regular telephone follow-up was conducted after discharge to timely answer relevant questions about prevention of CHD for patients and their family members [7–10].

Based on routine health education, patients in the research group received the community-family management mode under Internet MT monitoring. (1) Health education team for the research group: CHD health education team was jointly set up by the professional nurses and community nurses to first conduct intensive training with contents mainly involving the community-family management mode, CHD prevention, medication management, connection between Internet MT and health management mode, behavior restriction, and diet guidance. (2) Condition evaluation: patients took a physical exam in the community hospital every half a year, and their CHD condition, especially the risk factors for CHD, was evaluated by the nursing personnel; before implementing the community-family health management mode, the health profiles of all patients were created, mainly including their general information, health status, and condition analysis; the stable population and risk population were divided according to the results of each condition evaluation, the health education management was strengthened for the risk population, and the treatment modality was adjusted when necessary. (3) Making CHD health education manual: personalized health education manuals were made according to patients' age, living environment, family members' cognition of CHD, and daily diet, with contents mainly including basic knowledge of CHD, cause of disease, pathomechanism, treatment modality, diet guidance, exercise guidance, basic home care knowledge, and self-care knowledge [4, 11]. (4) Implementation of health education: health education lectures about CHD prevention and care including on-site demonstration were carried out, health education manuals were distributed at the community health service station, family members were encouraged to join the lecture, and at the end of the lectures, the nursing personnel timely answered the questions for patients and their family members and recorded the health education contents and their degree of grasp of the knowledge in the health profiles [12]. A mobile phone terminal information resource sharing platform based on Internet technology was established, which mainly contained four modules, patient information, individual consultation, CHD health knowledge, and patient communication, so that the nursing personnel in the health education team could carry out active online intervention to patients and their family members and conduct analysis of classic cases and communication on home care knowledge to patients and their family members via the community local network and WeChat group, and patients and their family members could consult the community nursing personnel at any time via the Internet terminal; in the form of setting up the WeChat official account, the nursing personnel timely pushed the knowledge of CHD prevention and care to patients and their family members, especially paying close attention to the health of high-risk population via the Internet platform.

### 2.4. Observation Indexes

(1) Patients' general data such as age, BMI, course of CHD, educational degree, symptom manifestations, and gender were recorded for statistic. (2) Six months after intervention, patients' blood pressure, blood glucose, triglyceride (TG), and total cholesterol (TC) level were measured at reexamination. (3) Patients' degree of grasp of CHD health knowledge was assessed by the CHD rehabilitation knowledge assessment scale [13] with Cronbach's *α* coefficient of 0.833, which contained 5 dimensions (exercise, diet, medication, basic knowledge, and risk factors) and 50 items; each item was rated by the 3-point scoring method on a scale of 0–2 points, and the score value was in direct ratio to their grasp of rehabilitation knowledge. Patients' living style, control of risk factors, and compliance with regular follow-up and medication were assessed by the secondary prevention behavior assessment scale, which had 25 items, with higher scores indicating better execution of secondary prevention behavior. (4) Patients' angina was assessed by the Seattle Angina Questionnaire (SAQ) [14], which covered physical limitation, anginal stability, anginal frequency, disease perception, and treatment satisfaction with total 20 items. After each item was scored, the standard score was calculated by the formula standard score = (actual score − lowest score)/(highest score − lowest score) × 100%, with higher scores indicating better somatic function. The scale had the total Cronbach's *α* coefficient of 0.759, with better reliability, validity, and responsibility. (5) The readmission of patients 1 year after intervention was counted. (6) Quality of life (QOL): patients' prognostic QOL was assessed by the Chinese Questionnaire on Quality of Life in Patients with Cardiovascular Disease (CQQC) [15] on a scale of 0–154 points, with higher scores indicating better QOL.

### 2.5. Statistical Processing

In this study, the between-group differences in data were processed by SPSS 22.0, the picture drawing software was GraphPad Prism 7 (GraphPad Software, San Diego, USA), the items included were enumeration data and measurement data, which were expressed by (*n*(%)) and ($\bar{X}$ ± *s*) and examined by the *X*^2^ test and *t*-test, respectively, and differences were considered statistically significant at *P* < 0.05.

## 3. Results

### 3.1. General Data

No statistical between-group differences in patients' age, BMI, course of CHD, educational degree, symptom manifestations, and gender were observed (*P* > 0.05), as given in Table 1.

### 3.2. Laboratory Indexes

Six months after intervention, the control of patients' blood pressure, blood glucose, TG, TC, and other laboratory indexes was obviously better in the research group than in the control group (*P* < 0.05), as given in Table 2.

### 3.3. Scores on Rehabilitation Knowledge Level and Secondary Prevention Behavior

After intervention, the scores on rehabilitation knowledge level and secondary prevention behavior were obviously higher in the research group than in the control group (*P* < 0.05), as shown in Figure 1.

### 3.4. SAQ Score

Six months after intervention, the scores on patients' physical limitation, anginal stability, anginal frequency, disease perception, and treatment satisfaction were obviously higher in the research group than in the control group (*P* < 0.05), as given in Table 3.

### 3.5. Readmission Rate

According to the statistical results shown in Figure 2, the readmission rate within 1 year of intervention was significantly lower in the research group than in the control group (*P* < 0.05).

### 3.6. QOL

The total score of CQQC and scores on physical strength, condition, general life, and social mentality were significantly better in the research group than in the control group (*P* < 0.05), as given in Table 4.

## 4. Discussion

According to the statistics of clinical data, CHD has become one of the diseases with the highest morbidity and mortality rate among residents in China, and more and more younger people suffer from CHD, so the prevention and treatment of CHD, rehabilitation, and health management have become the urgent issues [16–18]. The Chinese Experts Consensus on Cardiac Rehabilitation/Secondary Prevention for Coronary Artery Disease [19] proposed that CHD rehabilitation includes three phases, i.e., phase I rehabilitation (in-hospital rehabilitation), phase II rehabilitation (early out-of-hospital rehabilitation), and phase III rehabilitation (home rehabilitation), and the specific contents of cardiac rehabilitation are stressed in the phase III rehabilitation, including lifestyle changes (smoking cessation/diet/exercise), psychocardiology health (sleep management), evidence-based medication, QOL assessment and improvement, and occupational rehabilitation. The rehabilitation content of each rehabilitation stage has particular emphasis, and it can be seen that both community and home care interventions are important in the health management of CHD patients. With the continuous development of Internet technology, the products of mobile Internet devices, such as WeChat, apps, and miniprograms, also play an important carrier role in the health management of patients, so that the forms of health education gradually diversify, which creates more possibilities for the improvement of health management levels in CHD patients [20–23]. Therefore, a community-family management mode under Internet-based MT monitoring was established by our hospital to strengthen the intervention on patients' psychological status and adverse health behaviors, promote their body recovery, and improve their self-management ability.

A total of 86 patients with stable CHD treated in our hospital were screened as the study objects, and 43 of them who received the routine intervention were selected as the control, so as to retrospectively analyze the actual application effect of community-family management mode under Internet MT monitoring in elderly patients with CHD, and the study concluded that 6 months after intervention, the control of laboratory indexes including patients' blood pressure, blood glucose, TG, and TC was obviously better in the research group than in the control group (*P* < 0.05); after intervention, the scores on patients' rehabilitation knowledge level and secondary prevention behavior were obviously higher in the research group than in the control group (*P* < 0.05), which was consistent with the study by Guo et al. [24]; 6 months after intervention, patients' scores on physical limitation, anginal stability, anginal frequency, disease perception, and treatment satisfaction were obviously higher in the research group than in the control group (*P* < 0.05); within 1 year of intervention, the readmission rate was significantly lower in the research group than in the control group (*P* < 0.05); and the total score of CQQC and scores on physical strength, condition, general life, and social mentality were significantly better in the research group than in the control group (*P* < 0.05). The findings confirmed that the effective combination of Internet MT monitoring and community-family management mode can effectively control the condition of CHD patients and improve the disease perception of patients and their family members. This model achieved close integration of community and family, and at the same time, with the aid of modern science and technology, boosted the intensity of intervention for patients and made up for the drawbacks of the traditional preaching model, while enabling patients or their family members to receive corresponding nursing knowledge through mobile terminals, which was conducive to enhancing their self-care awareness. It is an effective continuation of clinical care, and the intervention of Internet MT greatly increases the application space of community-family management mode and makes health management content and intervention modalities more diverse, thereby promoting the improvement of disease and body recovery, as well as quality of life.

In summary, the community-family management mode under Internet-based MT monitoring is an effective continuation of clinical care for elderly patients with stable CHD, which has played an effective role in daily index monitoring of patients, stabilizing the condition, promoting patients' disease perception, reducing the readmission rate, and improving patients' prognostic QOL. However, according to some surveys, community health service resources in most regions of China cannot meet the increasing social demands, and thus, community healthcare workers are less confident in the prevention and treatment of CHD, resulting in the poor control of the disease in elderly patients. Therefore, it is necessary to further explore the content, methods, and forms of community supportive interventions in combination with the situation of community medical treatment.

## Figures and Tables

**Figure 1:** Statistics of scores on rehabilitation knowledge level and secondary prevention behavior of the two group. The horizontal axis indicates the assessment dimensions, and the vertical axis indicates the scores. Six months after intervention, the scores on rehabilitation knowledge level and secondary prevention behavior of the control group were, respectively, (70.05 ± 7.24) and (70.33 ± 8.52). Six months after intervention, the scores on rehabilitation knowledge level and secondary prevention behavior of the research group were, respectively, (86.12 ± 6.43) and (81.22 ± 6.15). ^*∗*^Significant difference in patients' rehabilitation knowledge level between the two groups (*t* = 10.883, *P* < 0.001). ^∗∗^Significant difference in patients' secondary prevention behavior between the two groups (*t* = 6.796, *P* < 0.001).

**Figure 2:** Statistics of readmission rate of the two groups within 1 year of intervention. The horizontal axis indicates the readmission rate, and the vertical axis indicates the percentage. The readmission rate within 1 year of intervention of the control group was 23 (43.49%). The readmission rate within 1 year of intervention of the research group was 10 (23.26%). ^*∗*^Significant difference in the readmission rate between the two groups (*X*^2^ = 8.310, *P*=0.004).

**Table 1:** Comparison of patients' general data between the two groups (*n* = 43).

Observation index	Control group	Research group	*X* ^2^/*t*	*P*
Age (years)	58.42 ± 3.57	57.88 ± 3.63	0.695	0.489
BMI (kg/m^2^)	24.11 ± 3.05	24.15 ± 3.02	0.061	0.951
Course of CHD				
≤1 year	8 (18.60)	7 (16.28)	0.387	0.534
1-2 years	12 (27.91)	14 (32.56)	0.221	0.639
≥2 years	23 (53.49)	22 (51.16)	0.047	0.829
Educational degree			0.195	0.659
Junior high school and below	25 (58.14)	27 (62.79)		
Senior high school	18 (41.86)	16 (37.21)		
Gender			0.199	0.655
Male	26 (60.47)	28 (65.12)		
Female	17 (39.53)	15 (34.88)		
Symptom manifestation				
Angina	20 (46.51)	21 (48.84)	0.047	0.829
Myocardial sclerosis	15 (34.88)	17 (39.53)	0.199	0.655
No symptom	8 (18.60)	5 (11.63)	0.816	0.366

**Table 2:** Statistics of laboratory indexes of patients in the two groups 6 months after intervention.

Test indicator	Control group	Research group	*t*	*P*
Blood pressure (mmHg)				
Systolic blood pressure	121.75 ± 6.40	117.86 ± 5.30	3.70	0.003
Diastolic blood pressure	83.05 ± 4.03	73.25 ± 3.61	11.878	<0.001
Fasting blood glucose (mmol/L)	7.06 ± 1.30	6.02 ± 1.17	3.899	<0.001
TG (mmol/L)	1.64 ± 0.58	1.21 ± 0.37	4.099	<0.001
TC (mmol/L)	4.13 ± 0.55	3.42 ± 0.34	7.200	<0.001

**Table 3:** Statistics of SAQ scores of the two groups.

Evaluation dimension	Control group	Research group	*t*	*P*
Physical limitation	69.88 ± 8.71	77.41 ± 6.22	4.613	<0.001
Anginal stability	72.72 ± 10.82	81.06 ± 6.08	4.406	<0.001
Anginal frequency	63.22 ± 7.61	72.10 ± 6.25	5.913	<0.001
Disease perception	63.71 ± 8.55	78.26 ± 7.10	8.585	<0.001
Treatment satisfaction	74.35 ± 7.42	88.32 ± 6.09	9.543	<0.001

**Table 4:** Statistics of CQQC scores of the two groups.

Assessment item	Control group	Research group	*t*	*P*
Total score	95.88 ± 10.24	120.14 ± 11.34	10.412	<0.001
Physical strength	28.13 ± 4.85	33.05 ± 5.18	4.547	<0.001
Condition	22.13 ± 3.24	27.15 ± 4.56	5.885	<0.001
General life	17.81 ± 2.80	21.34 ± 2.17	6.534	<0.001
Social mentality	18.19 ± 3.07	26.13 ± 3.15	11.837	<0.001

## Data Availability

The data used to support the findings of this study are available from the corresponding author upon request.
